This article has been retracted.

# Image Segmentation Technology Based on Attention Mechanism and ENet

**DOI:** 10.1155/2022/9873777

**Published:** 2022-08-04

**Authors:** Ling Ma, Xiaomao Hou, Zhi Gong

**Affiliations:** School of Computer Science and Engineering, Hunan University of Information Technology, Changsha 410151, Hunan, China

## Abstract

With the development of today's society, medical technology is becoming more and more important in people's daily diagnosis and treatment and the number of computed tomography (CT) images and MRI images is also increasing. It is difficult to meet today's needs for segmentation and recognition of medical images by manpower alone. Therefore, the use of computer technology for automatic segmentation has received extensive attention from researchers. We design a tooth CT image segmentation method combining attention mechanism and ENet. First, dilated convolution is used with the spatial information path, with a small downsampling factor to preserve the resolution of the image. Second, an attention mechanism is added to the segmentation network based on CT image features to improve the accuracy of segmentation. Then, the designed feature fusion module obtains the segmentation result of the tooth CT image. It was verified on tooth CT image dataset published by West China Hospital, and the average intersection ratio and accuracy were used as the metric. The results show that, on the dataset of West China Hospital, Mean Intersection over Union (MIOU) and accuracy are 83.47% and 95.28%, respectively, which are 3.3% and 8.09% higher than the traditional model. Compared with the multiple watershed algorithm, the Chan–Vese segmentation algorithm, and the graph cut segmentation algorithm, our algorithm increases the calculation time by 56.52%, 91.52%, and 62.96%, respectively. It can be seen that our algorithm has obvious advantages in MIOU, accuracy, and calculation time.

## 1. Introduction

Since the 1970s, with the rapid development of computer technology, all walks of life have undergone tremendous changes [1]. The application of computer imaging technology in the medical field has made great progress in medical imaging technologies such as ultrasound detection, electroencephalography, magnetic resonance imaging (MRI), and CT. It is applied to many subjects such as brain surgery, cardiothoracic surgery, orthopedics, and stomatology, which greatly improves the accuracy of modern medical diagnosis and also improves people's physical health and quality of life [2–4].

Medical images produced by different imaging technologies have different characteristics. For example, both CT and MRI images give anatomical information of target, but MRI is better at distinguishing soft tissues with similar densities such as gray matter and white matter in the brain tissue. CT images are better in areas with large differences in the density of bone tissues [5, 6]. Nevertheless, the continuous two-dimensional slice image set provided by these devices can only intuitively receive certain section information of a certain part of the organ, and it is easy to get tired. The interpretation of these image sequences requires doctors to have excellent three-dimensional space imagination capabilities, rich clinical experience, and accurate professionalism, which increases medical costs. Therefore, some researchers use image segmentation technology to extract feature points in the image and perform region segmentation. Later, using visualization technology, the medical image sequence is transformed into a three-dimensional space model and the slice data are visually displayed to the medical staff. It can quickly and accurately perform multidirectional and multilevel observation of the patient's slice data, which greatly reduces the clinical cost and improves the treatment efficiency [7–9].

With the rapid development of GPU update iterations, the application of neural networks has become more widespread and it has become possible for medical images to be processed by neural networks [10]. Neural network technology is developed from machine learning. After people input the sample image and the corresponding label to the computer, the computer searches for the characteristic mark corresponding to the image. Image data will have to produce different data results through operations such as convolution and pooling. These results will be compared with the label to generate corresponding feedback. The result that conforms to the label strengthens the corresponding weight in the neural network process through the reverse transfer process, and vice versa, reduces the weight. Repeat this process until the loss value reaches your expectations, which is the neural network model training process [11–13]. After the training is completed, the weights of each part of the network are randomly determined and no longer change with the input of image data. Input the test set into the trained network model, the model will predict the image according to the network weight of each layer and give a probability map [14]. It is used to express the probability of each area of the image as the target and finally output the segmentation result. This process is model prediction. The existing image segmentation technology has low robustness when processing medical images and has poor matching ability for soft tissues (such as internal organs) with inconspicuous grayscale intervals and hard tissues (such as teeth) with small structural gaps. Edge prediction is also unsatisfactory [15].

Modern medical CT scans mainly include multiple spiral computed tomography (MSCT) and cone beam computed tomography (CBCT). CBCT is more commonly used in dentistry, which has characteristics of short scanning time and low radiation dose [16]. Because the bones of the teeth and some soft tissues are closely intertwined in the CT scan of the tooth, the boundary of the CT image will become very blurred. Not only the CT images of teeth but also the CT images of various organs have this problem more or less. This is the first problem that needs to be solved [17]. To reduce radiation impact on body, CBCT reduces the scanning time and radiation dose. This causes adhesions between adjacent teeth in the crown of the tooth in the CT image. The tooth gap is small, the contrast between the root and the alveolar bone is low, and the gray value distribution between the teeth is also different. There may also be differences in gray values of the same tooth, and the topological structure is more complicated and not easy to distinguish. This is the most important problem to be solved in tooth segmentation in medical images [18–20].

The remaining chapters of this paper are arranged as follows: Section 2 introduces the related research; Section 3 introduces the theory and methods used in this paper in detail; Section 4 verifies the performance of the model through experiments and analyzes the results; Section 5 is the paper conclusion.

## 2. Related Research

In recent years, level set algorithms are often used in medical image processing with complex curve topologies. Osher et al. [21] proposed a level set method based on the geometric deformation model to solve the topological structure change problem in curve evolution that cannot be solved by previous algorithms. Due to its good working efficiency, this algorithm is applied in many fields. Huang et al. [22] used the level set function to partition MRI images. The energy function is constructed with variable differentiation, which improves its accuracy and robustness to a certain extent. Yang et al. [23] added Markov random field (MRF) to the level set method to establish the correlation between pixels and their neighboring areas to reduce calculations and enhance the robustness of the algorithm. However, the problem of the amount of calculation has not been fully resolved. Mansouri et al. [24] involved the level set method in machine learning to segment cardiac MRI images and expected to use the computing power of machine learning to accelerate the level set solution. However, in the end, complete edge details cannot be obtained.

At present, thanks to the improvement of backpropagation algorithms, neural networks stand out in machine learning. Among them, the convolutional neural network (CNN) has the most far-reaching influence and has attracted much attention. He et al. [25] used the residual network to map the output of previous layer to the following results to supplement the lack of high-level information after multiple trainings. Alom et al. [26] replaced the original U-Net submodules with residual networks and recurrent neural networks. Yao et al. [27] proposed focused convolution for semantic segmentation, adding neural network multiscale processing capabilities. Mondal et al. [28] used adversarial learning mechanism for semisupervised segmentation to combat overfitting. Qi et al. [29] used an unsupervised way to align the features of the target area. Liu et al. [30] used the RNN network for lesion segmentation, enhanced the detailed information of the target area, and realized the recognition of small features of medical images.

Most of the above studies did not consider the close interweaving of tooth bones and some soft tissues, which will cause the image boundary of the tooth CT to become very blurred. Aiming at the particularity of tooth CT images, a tooth CT image segmentation network combined with attention mechanism was constructed.

## 3. Theory and Method

### 3.1. ENet Network Architecture

Commonly used semantic segmentation algorithms such as FCN or SegNet are based on the VGG architecture, which requires a lot of floating-point operations and is of low timeliness. In response to this problem, a new type of encoder-decoder algorithm ENet algorithm emerged [31]. The algorithm optimizes the network model, reduces the number of network parameters while maintaining the accuracy of the model, and shortens the forward reasoning time. Based on these, we combine the ENet network with the attention mechanism and propose a tooth CT image segmentation method.

ENet is a lightweight network that uses a small number of models and parameters and is designed for low-latency manipulation tasks.  Figure 1 is a schematic diagram of the initialization operation of ENet. In CNN, with the increase in the number of layers, the vanishing gradient or the gradient explodes during the backpropagation process. Therefore, the initialization of the weights is very important. The left and right sides use a convolution with a step of 2 and a 2 × 2 maximum pooling to downsample the input image. Finally, the results of the two sides are combined through the Concat layer so that the size of the feature map is reduced to half of the original after the initialization module, which reduces the size of the overall model.

The ENet algorithm introduced the bottleneck structure for the first time. Different bottleneck structures represent different functions. Each bottleneck is composed of a main line and an auxiliary line in order to learn the residuals. In the encoder stage, there are mainly two types of bottleneck: one is the downsampling bottleneck that includes the pooling layer and the other is the basic bottleneck for feature extraction. The structure is shown in Figure 2. In downsampling bottleneck, the main line is composed of three convolutional layers. First, a 2 × 2 convolution (step size 2) is used for a downsampling, and then an ordinary convolution is performed to extract features. The convolution method can be selected from ordinary convolution, decomposition convolution, and hole convolution according to different functions. Finally, a 1 × 1 convolution kernel is used for feature enhancement. After each convolution, a normalization layer BatchNorm and activation function PReLU are connected. The auxiliary line consists of a maximum pooling layer and a 1 × 1 convolutional layer. Maximum pooling is responsible for extracting context information. The role of the convolutional layer is channel conversion so that the number of characteristic channels is consistent with the main line, which is convenient for fusion with the main line through the Eltwise layer. In the basic feature module, the main line is similar to the downsampling module. A 1 × 1 projected convolutional layer, a common convolutional layer for feature extraction, and a 1 × 1 convolutional layer for dimension enhancement are sequentially passed through. The auxiliary line is directly superimposed on the main line through the Eltwise layer with an identity mapping.

The overall architecture of ENet is shown in Table 1. The ENet algorithm greatly reduces the overall calculation amount and parameter amount through the early downsampling and decomposition convolution of the network, which improves the real-time performance of the network. However, the design of the network is to accelerate the reasoning of the network and ignore the impact on accuracy. Therefore, the image segmentation effect of the ENet algorithm is not good.

### 3.2. Attention Mechanism Module

As only the ENet algorithm is used, the real-time performance of the network is mainly improved. However, the design of the network is to accelerate the reasoning of the network and ignore the impact on accuracy. Therefore, we added the attention module to improve network accuracy. In view of human attention mechanism, deep learning attention mechanism is essentially a tendentious resource allocation mechanism. Attention mechanism makes the network focus on the region with the most abundant information rather than the whole image in the classification process. Attention mechanism is an analysis technology to solve the problems in the fields of image recognition, speech signal recognition, natural language processing, and so on. Its principle stems from the selective attention mechanism of human visual system. The human visual system can quickly scan the whole image and quickly locate the expected main area, that is, first understand the whole picture and then focus on the key points. The combination of face and point can identify things more accurately and quickly. The feature extraction part of the attention module built in this paper is shown in Figure 3.

First, the global average pooling is used to change the data output from the dense layer from *W* × *H* × K to 1 × 1 × *K*.

(1) $$\begin{array}{c} Z_{c}=F_{sq}\left(u_{c}\right)\frac{1}{H\times W}\sum_{i=1}^{H}\sum_{j=1}^{W}u_{c}\left(i,j\right), \end{array}$$

where *F*_*sq*_ is the global average pooling function.

Next, perform two FC operations on the network. *C* is the dimensionality reduction coefficient. The experiment shows that the best performance is obtained when *C* = 16. The equation is as follows:

(2) $$\begin{array}{c} s=F_{ex}\left(z,W\right)=\sigma \left(g\left(z,W\right)\right)=\sigma \left(W_{2}\delta \left(W_{1}z\right)\right), \end{array}$$

where *σ* and *δ* represent sigmoid and ReLU activation functions, respectively, and *W*_1_, *W*_2_ ∈ *R*^*K*^2^/*C*^.

Then, perform the scale operation to change the data into *W* × *H* × K.

(3) $$\begin{array}{c} X_{c}=F_{\text{scale}}\left(u_{c},s_{c}\right)=u_{c}\cdot s_{c}. \end{array}$$

When the attention module is not added to the network, the batch size is 256 and the size is 224 × 224, and the time of one forward propagation is 42 ms. After adding the attention module, the elapsed time is 47 ms. After reducing the complexity by changing the network dimension, the consumption time still increases slightly, but compared with the improvement of segmentation accuracy, this can be completely ignored.

In addition, the skip connection in the network in this paper is not the same as DenesNet [32]. DenesNet only has connections in the blocks between downsampling, whereas our network has connections in all layers. In the pooling method, this paper adopts atrous spatial pyramid pooling (ASPP). Global context is augmented by combining image features with GAP. It consists of four parallel operations, one 1 × 1 convolution and three 3 × 3 convolutions, with batch normalization added.

## 4. Experimental Results and Analysis

### 4.1. Experimental Environment and Network Parameters

The dataset used in the experiment in this section is provided by West China Hospital. The algorithm experiment in this article is based on the Keras framework. The framework is developed by Google and uses TensorFlow and Theano to package and integrate many basic neural network structures and some mature algorithms. The experimental dataset used is dental CT data provided by West China Hospital. The CPU is an 8 GB Intel Core i7-6700, and the GPU is NVIDIA GeForce GTX 1070.

During training, the optimization method uses stochastic gradient descent. The momentum parameter is set to 0.9, initial learning rate is 8 × 10^−3^, and weight decay rate is 1 × 10^−4^. In order to increase the generalization ability, the dataset adopts data augmentation. Using random horizontal flips and 0–2 pixel translation on the input image axis increases the training dataset. Before entering network, normalized image gray value is [0 ∼ 1] and image size is 512 × 512. Our original data have 400 images. Among them, there are 300 images in the training set and 100 images in the validation set. After data augmentation, our training set has 1500 images and the validation set has 500 images. The K-fold cross-validation technique was used during training, where *K* = 10.

The comparison effect between the labeled CT image data and the original image is shown in Figure 4.

### 4.2. Evaluation Index

We use two metrics to evaluate the accuracy of the tooth CT image segmentation algorithm. The pixel accuracy (PA) formula is as follows:

(4) $$\begin{array}{c} \text{PA}=\frac{\sum_{i=0}^{k}p_{ii}}{\sum_{i=0}^{k}\sum_{j=0}^{k}p_{ij}}. \end{array}$$

Among them, *p*_*ii*_ is the correct number of divisions, *p*_*ij*_ is the number of pixels that originally belonged to category *i* but were divided into category *j*, and *p*_*ji*_ is the number of pixels that originally belonged to category *j* but were divided into category *i*. There are *k* + 1 categories.

The calculation formula of MIOU is as follows:

(5) $$\begin{array}{c} \text{MIOU}=\frac{1}{k+1}\sum_{i=0}^{k}\frac{p_{ii}}{\sum_{j=0}^{k}p_{ij}+\sum_{j=0}^{k}p_{ji}-p_{ii}}. \end{array}$$

Our experiment stops training after 80 epochs, and the change curves of MIOU, PA, and loss of the validation set during training are described in Figure 5.

The MIOU value reached 80% when network was trained to the 20th epoch. It can be seen that the performance of our network is very good and the follow-up is also relatively stable. From the perspective of quantitative indicators, the expected results have been achieved.

### 4.3. Algorithm Effect Comparison

After the feature map of the segmented image is obtained, the pixel-by-pixel probability prediction is performed on it and the classification probability map of the image region is obtained. Then, the pixels are classified and divided according to these probability maps. The pixels of the same type are converted into a region to get image segmentation result. It is described in Figure 6.

In Figure 6, the leftmost column is the original CT image of tooth. The middle column is the segmentation result of this algorithm. The column on right is the segmentation result of U-Net algorithm. It can be found from Figure 5 that our algorithm can effectively segment the tooth CT image. The effect of tooth edge extraction is better than U-Net, but there is still some noise influence. There is a certain shadow in the center of the segmentation result, but there is no shadow in U-Net. The objective data of the algorithm in this paper, FCN, and U-Net are shown in Figure 7.

Figure 7 shows comparison between our algorithm and other two semantic segmentation algorithms. All three comparison methods are trained on the same dataset and get test results. The number of test set images used to compare our algorithm with other algorithms is 300. Among them, the weight decay rate for training U-Net and FCN is 1 × 10^−4^, initial learning rate is 8 × 10^−3^, momentum parameter is set to 0.9, and training batch size is 20. The training time was 12 hours and 10 hours, respectively. It can be seen that our algorithm is superior to the FCN network in MIOU and time. Our algorithm is slightly lower than that of U-Net in MIOU, and the training speed of our algorithm is obviously better than that of U-Net in terms of segmentation time. The results show that our algorithm can effectively speed up the computation of the model while ensuring high segmentation accuracy.

Our algorithm can perform relatively accurate feature extraction on tooth CT images, thereby accurately segmenting. The pixel-by-pixel prediction can well deal with the adhesion problem in the tooth CT image. In terms of segmentation results and computing speed, our algorithm is compared and evaluated with algorithms such as graph cut. The final results of each algorithm are shown in Figure 8.

This article uses multiple sets of images of the dataset provided by Huaxi to conduct experiments. Figure 8 shows results obtained on part of validation set. The first column of Figure 8 is the original image of the input image, the second column is segmentation result of this algorithm, the third column is segmentation result of multiple watershed algorithm, the fourth column is segmentation result of Chan–Vese model, and the fifth column is graph cut algorithm. Our method has the best segmentation accuracy. The result of comparing MIOU and speed is shown in Figure 9.

Figure 9 shows the results of multiple watershed algorithm [6], Chan–Vese segmentation algorithm [25], graph cut segmentation algorithm [3], and the algorithm in this paper on the test set. It shows that the neural network model has a well effect in image segmentation. The MIOU of graph cut is close to the algorithm in this article, but the graph cut algorithm can only process one image at a time. Also, each segmentation needs to manually draw 3–5 lines to divide the area, which is difficult to achieve automatic segmentation. In terms of computing speed, the algorithm in this paper uses a neural network framework to averagely segment an image in one second. If graph cut does not calculate the time of manual scribing, each image is processed for an average of 2.7 seconds. The Chan–Vese algorithm must complete the specified number of iterations regardless of whether the curve evolution is already in an oscillating state during the process. The relevant parameters of the Chan–Vese algorithm are set as follows: epison = 1, step = 1, and LSF = IniLSF. On average, an image takes 11.8 seconds. The multiple watershed method takes 2.3 seconds to process an image on average. It can be known that our algorithm is better than traditional methods.

## 5. Conclusion

We propose a semantic segmentation algorithm for dental CT images. The ENet, which has both segmentation speed and accuracy, is used as the backbone network. At the same time, an attention mechanism is added to make the network improve the weight of useful information. Also, a feature fusion module is constructed to integrate the features of different receptive fields, thereby improving the segmentation accuracy. Our method is tested on the public tooth CT image dataset in West China, and the final result is compared with a variety of algorithms. The results show that, on the dataset of West China Hospital, Mean Intersection over Union (MIOU) and accuracy are 83.47% and 95.28%, respectively, which are 3.3% and 8.09% higher than the traditional model. Our algorithm has achieved better results. Next, the attention mechanism module will be further improved. How to more effectively improve the accuracy and speed of tooth segmentation so that it can be directly applied to the clinic is our next research direction.

## Figures and Tables

**Figure 1:** Initialization operation.

**Figure 2:** Schematic diagram of different bottleneck structures: (a) downsampling bottleneck; (b) basic bottleneck.

**Figure 3:** Feature extraction module.

**Figure 4:** Original images and labeled images.

**Figure 5:** Curves of MIOU, PA, and loss.

**Figure 6:** Comparison between our algorithm and the U-Net segmentation model.

**Figure 7:** Comparison of our algorithm with other methods.

**Figure 8:** Comparison of our algorithm with other algorithms.

**Figure 9:** Comparison of our algorithm with other algorithms.

**Table 1:** Framework of ENet.

	Name	Type	Output size
	Initial		16 × 256 × 256

1	Bottleneck	Downsampling	64 × 128 × 128
	4 × Bottleneck 1		64 × 128 × 128

2	Bottleneck 2.0	Downsampling	128 × 64 × 64
	Bottleneck 2.1		128 × 64 × 64
	Bottleneck 2.2	Dilated 2	128 × 64 × 64
	Bottleneck 2.3	Asymmetric 5	128 × 64 × 64
	Bottleneck 2.4	Dilated 2	128 × 64 × 64
	Bottleneck 2.5		128 × 64 × 64
	Bottleneck 2.6	Dilated 2	128 × 64 × 64
	Bottleneck 2.7	Asymmetric 5	128 × 64 × 64
	Bottleneck 2.8	Dilated 16	128 × 64 × 64

3	Repeat section 2	Without bottleneck 2.0	

4	Bottleneck 4.0	Upsampling	64 × 128 × 128
	Bottleneck 4.1		64 × 128 × 128
	Bottleneck 4.2		64 × 128 × 128

5	Bottleneck 5.0	Upsampling	16 × 256 × 256
	Bottleneck 5.1	Upsampling	16 × 256 × 256
	FC		*C* × 512 × 512

## Data Availability

The data used to support the findings of this study are included within the article.
